The article "LncRNA SNHG3 enhances the malignant progress of glioma through silencing KLF2 and p21" was retracted in 2021. Reasons: manipulated images; duplicated images; concerns about the images.

# LncRNA SNHG3 enhances the malignant progress of glioma through silencing KLF2 and p21

**DOI:** 10.1042/BSR20180420

**Published:** 2018-09-07

**Authors:** Fan Fei, Yongsheng He, Sen He, Zhongze He, Youyu Wang, Gang Wu, Mengni Li

**Affiliations:** 1 Department of Neurosurgery, Hospital of The University of Electronic Science and Technology of China and Sichuan Provincial People’s Hospital, No.32 West Second Section First Ring Road, Chengdu 610072, Sichuan, China; 2 Department of Neurosurgery, Graduate School of Zunyi Medical University, Zunyi 563003, Guizhou, China; 3 Department of Thoracic Surgery, Hospital of The University of Electronic Science and Technology of China and Sichuan Provincial People’s Hospital, No.32 West Second Section First Ring Road, Chengdu 610072, Sichuan, China; 4 Department of Hepatobiliary surgery, Hospital of The University of Electronic Science and Technology of China and Sichuan Provincial People’s Hospital, No.32 West Second Section First Ring Road, Chengdu 610072, Sichuan, China; 5 Department of Pediatrics, Hospital of The University of Electronic Science and Technology of China and Sichuan Provincial People’s Hospital, No.32 West Second Section First Ring Road, Chengdu 610072, Sichuan, China

**Keywords:** glioma, KLF2, p21, SNHG3

## Abstract

As a newly discovered long non-coding RNA, small nucleolar RNA host gene 3 (SHNG3) has been reported to be dysregulated in certain cancers. Nevertheless, the details about clinical values and biological effects of SNHG3 on glioma are still covered. In this paper, we determined the expression level of SNHG3 in glioma tissues and cells and evaluated the effect of SNHG3 expression on the prognosis of glioma patients. The functional assays were applied to define the effects of SNHG3 on the biological behaviors in glioma including cell proliferation, cell cycle, and apoptosis. It was revealed that SNHG3 was much more enriched in glioma tissues and cell lines than in normal ones. Furthermore, gain- or loss-of-function experiments indicated that the up-regulation of SNHG3 promoted cell proliferation, accelerate cell cycle progress, and repressed cell apoptosis. The mechanistic assays disclosed that SNHG3 facilitated the malignant progression of glioma through epigenetically repressing KLF2 and p21 via recruiting enhancer of zeste homolog 2 to the promoter of KLF2 and p21. Generally, it was exposed that SNHG3 might function as an oncogene in glioma and could be explored as a potential prognostic biomarker and therapeutic target for glioma.

## Introduction

As one of the commonest types of main brain tumor for adults, glioma represents one of the most fateful cancers for human [1]. Although great progress has been made in glioma treatment, including surgery, chemotherapy, and radiotherapy, the clinical prognosis for glioma patients is still unsatisfied [2,3]. Thus, it is critically important to figure out the molecular mechanisms engaged in the initiation and development of glioma. It will benefit the patients greatly to confirm underlying biomarkers and therapeutic targets.

On the basis of the genome sequencing technology, it was clarified that only ~2% of the mammalian genome is capable of encoding proteins, while the rest belongs to non-protein-coding RNAs (ncRNAs) [4]. As one member of the ncRNAs, long non-coding RNAs (lncRNAs) have more than 200 nt and participate in various biological modifications including epigenetic modification, transcriptional, or post-transcriptional regulation [5,6]. Accumulative lncRNAs have been discovered to be associated with the progression of tumors, such as lncRNA H19 in melanoma [7], lncRNA CAF in oral squamous cell carcinoma [8], and lncRNA XIST in lung cancer [9]. In addition, there are also many reports about the roles of lncRNAs in glioma. For instance, lncRNA HOXA11-AS, MALT1 and CRNDE, and so on in glioma [10–12]. As a newly discovered lncRNA, small nucleolar RNA host gene 3 (SHNG3) has just been discussed in colorectal cancer and hepatocellular carcinoma [13,14]. Here, it was discovered that SNHG3 was more highly expressed in glioma tissues, especially in tissues with advanced tumor grade, and cell lines. Furthermore, high expression of SNHG3 predicted poor prognosis for patients. Subsequently, functional assays exposed that silenced SNHG3 inhibited cell viability and proliferation, induced cell cycle arrest and apoptosis. The opposite results were obtained and observed after SNHG3 was overexpressed in U251 cells. Besides, it was also found out that KLF2 and p21 were down-regulated in glioma tissues. Spearman’s correlation analysis demonstrated the negative correlation among SNHG3, p21, and KLF2, confirmed again by qRT-PCR and Western blot rescue assays. Subcellular fractionation assay determined that SNHG3 was mainly located in nucleus. RIP and ChIP experiments disclosed that SNHG3 could sponge with enhancer of zeste homolog 2 (EZH2), while EZH2 was enriched in the promoters of KLF2 and p21, indicating the SNHG3-mediated and EZH2-induced HEK27me3 in the promoter regions of KLF2 and p21. In brief, SNHG3 facilitated the malignant progression of glioma through epigenetically repressing KLF2 and p21 via recruiting EZH2 to the promoter of KLF2 and p21.

## Materials and methods

### Patients’ samples

Sixty pairs of glioma tissue specimens and the matched adjacent healthy tissues were provided by Hospital of the University of Electronic Science and Technology of China and Sichuan Provincial People’s Hospital. All patients’ tissue specimens were promptly frozen in liquid nitrogen and maintained at −80°C for the isolation of RNA and proteins later. No patients had ever received any treatment from neurosurgery, chemotherapy, or radiotherapy. On the basis of WHO classification, all patients were classified into four histopathological grades: grade I, II, III, and IV. The present study had won the ethical approval from the Ethics Committee of Hospital of the University of Electronic Science and Technology of China and Sichuan Provincial People’s Hospital, and written informed consents had also been offered by each patient.

### Cell lines and culture

Four glioma cell lines (A172, U251, U87, and SHG44) were purchased from Shanghai Cell Bank of the Chinese Academy of Sciences (Shanghai, China), while the normal glial HEB cell was provided by American Type Culture Collection (ATCC; Manassas, VA, U.S.A.). The cells were cultivated in Dulbecco’s modified Eagle’s medium complemented with 10% of fetal bovine serum (Gibco; Thermo Fisher Scientific, Inc., Waltham, MA, U.S.A.). All cells were conserved in a humidified environment with 5% of CO_2_ at 37°C.

### Cell transfection

The short hairpin RNA used to target SNHG3, KLF2, and p21 was purchased from GenePharma (Shanghai, China). For the construction of SNHG3, KLF2 and p21 vectors, full-length HOTAIR was amplified and embedded into pcDNA3.1 vectors (Invitrogen, U.S.A.); and full open reading frame cDNA clones for KLF2 and p21 were transcribed, followed by the amplification of the products. Then, the DNAs were inserted into pcDNA3.1. The pcDNA3.0-SNHG3 and pcDNA3.0-KLF2 or pcDNA3.0-p21 vector plasmids were transfected into glioma cells using Lipofectamine 2000 (Invitrogen) in accordance with the manufacturer’s guidelines. Finally, glioma cell lines were transfected with oligonucleotides and constructs with Lipofectamine 2000 (Invitrogen, U.S.A.) on the basis of the manufacturer’s guidelines.

### RNA extraction and qRT-PCR

RNA was extracted from cells or tissues by using TRIzol (Invitrogen, U.S.A.), based on the manufacturer’s suggestions. qRT-PCR was used to measure the expressions of SNHG3, KLF2, and p21. The primers used in this process were listed as: SNHG3 (forward): 5′-TTCAAGCGATTCTCGTGCC-3′ and (reverse): 5′-AAGATTGTCAAACCCTCCCTGT-3′; KLF2 (forward): 5′-TTCGGTCTCTTCGACGACG-3′ and (reverse): 5′-TGCGAACTCTTGGTGTAGGTC-3′; p21 (forward): 5′-CAGCAGAGGAAGACCATGTG-3′ and (reverse): 5′-GGCGTTTGGAGTGGTAGAAA-3′; GAPDH (forward): 5′-GAAGAGAGAGACCCTCACGCTG-3′ and (reverse): 5′-ACTGTGAGGAGGGGAGATTCAGT-3′. Reverse transcription (RT) was performed by using Fermentas reverse transcription reagents and the Applied Biosystems^®^ TaqMan^®^ MicroRNA Reverse Transcription Kit (AppliedBiosystems, CA). The ABI StepOnePlus system (Applied Biosystems, CA) was applied to conduct the amplification reactions in accordance with the predetermined conditions. To evaluate the expression of SNHG3, GAPDH was applied for normalization. Data were analyzed by using the 2^–ΔΔ*C*^_t_ method. Each experiment was carried out for three times independently.

### Cell proliferation assays

A172 and SHG44 cells (4000 cells/well) were sealed in 96-well plates and cultured for 1, 2, 3, 4, or 5 days at 37°C, followed by the supplement of 10 μl of MTT solution (5 mg/ml) into each well within the appointed time. Fours hours later, the precipitates were dissolved by adding 200 μl of dimethyl sulfoxide into each well. Then, a micro-plate reader (Bio Tek Instruments, Inc., Winooski, VT, U.S.A.) was used to measure the absorbance value at 490 nm.

### Flow cytometry analyses

To analyze cell cycle, A172 and SHG44 cells were collected, fixed in 70% of ethanol, and stained with propidium iodide solution. Next, the FACSCalibur system (BD Biosciences) and FlowJo software (Tree Star Corp, Ashland, OR, U.S.A.) were used to analyze the flow cytometry images of the cell cycle. To observe cell apoptosis changes, cells (1 × 10^6^ cells/ml) were digested, decentralized, centrifuged, collected, washed with cold PBS, and resuspended in the binding buffer. Later, the cells were stained doubly with the phosphatidylethanolamine (PE) and annexin-V-FITC staining kit (BD Bio-sciences).

### Western blot

RIPA buffer (KenGEN, China) was used to isolate proteins from glioma cells or tissues. The BCA Protein Assay Kit (Beyotime, China) was applied to quantify the protein concentrations. Protein was split by 10% of SDS-PAGE, followed by the transferring onto PVDF membranes (Millipore, Billerica, MA, U.S.A.). The membranes were blocked with 5% of skim milk for 2 h. Subsequently, the membranes were cultivated overnight at 4°C with diluted antibodies against KLF2 and p21 (1: 1,000, Abcam, U.S.A.), followed by the culture with an HRP-conjugated secondary antibody (1:5000, YIFEIXUE BIO TECH, Nanjing, Jiangsu, China). GAPDH was used as a control (1:1000, YIFEIXUE BIO TECH, Nanjing, Jiangsu, China).

### Subcellular fractionation location

PARIS Kit (Life Technologies) was used to separate nuclear and cytoplasmic parts in accordance with the manufacturer’s suggestions. Briefly, 107 freshly cultivated glioma cells were collected, washed once in PBS, and then kept on ice. Next, cells were resuspended in the 100–500 μl of cell fractionation buffer and cultured on ice for 5–10 min. Specimens were centrifuged for 1–5 min at 4°C and 500 ***g***. The cytoplasmic fraction was aspirated away from the nuclear pellet that was washed in the ice-cold cell fractionation buffer, while the nuclear pellet was lysed in cell disruption buffer and the sample was separated to isolate RNA. The lysate was mixed with an equal volume of 2× Lysis/Binding Solution for RNA isolation; 1 ‘sample volume’ of 100% ethanol was added to the mixture and then washed with wash solution that was used to elute RNA. RNAs isolated from each of the fractions were analyzed by RT-qPCR to demonstrate the levels of nuclear-control transcript (U6), cytoplasm-control transcript (GAPDH), SNHG3.

### RNA immunoprecipitation (RIP)

RNA immunoprecipitation (RIP) experiments were performed with Magna RIP™RNA-Binding Protein Immunoprecipitation Kit (Millipore, U.S.A.), on the basis of the manufacturer’s guidance. The antibodies, EZH2, LSD1, for the RIP assays were purchased from Abcam. The total RNAs were the input controls.

### Chromatin immunoprecipitation

In order to generate DNA–protein cross-links, A172 and SHG44 cells were treated with formaldehyde and then were cultured for 10 min. Cell lysates were then sonicated to produce chromatin fragments of 200–300 bp, and then were immunoprecipitated with EZH2 and H3K27me3-specific antibody (Cell Signaling Technology) or IgG as control. Precipitated chromatin DNA was recovered and analyzed by qPCR.

### Statistical analysis

All data were shown as the mean ± standard deviation (SD) from three independent experiments. SPSS 18.0 software and GraphPad Prism 5.0 were used to perform statistical analyses. Differences among groups were determined by applying Student’s *t* test or one-way ANOVA analysis. A chi-square test was carried out to detect the relationship between the expression of SNHG3 and clinicopathological features. Cox regression analyses were used to analyze the independent prognostic importance of SNHG3. Kaplan–Meier method and log rank test were utilized to analyze the relevance between SHNG3 and the overall survival of glioma patients. *P*<0.05 was considered statistically significant.

## Results

### Highly expressed SNHG3 in glioma tissues and cells predicts poor prognosis

SHNG3 is a newly discovered lncRNA. In order to figure out the effect of SNHG3 on the initiation and development of glioma, we detected the expression of SNHG3 in glioma samples of TCGA database. It is obviously up-regulated in glioma samples than that in non-tumor tissue samples (Figure 1A). Furthermore, we detected the expression level of SNHG3 in 60 pairs of glioma tissues and non-malignant tissues. Unsurprisingly, the expression level of SNHG3 was higher in glioma tissues than that in non-tumor tissues (Figure 1B). In addition, the expression of SNHG3 in tissues with advanced stage was also significantly higher than that in early stage tissues (Figure 1C). The high expression of SNHG3 was also observed in glioma cell lines, compared with the normal cell (Figure 1D). According to the mean value of SNHG3 expression, glioma samples were divided into two group (SNHG3 high expression and SNHG3 low expression). Subsequently, high expression of SNHG3 was uncovered to be closely associated with KPS and tumor grade (Table 1). According to the result of Cox regression analysis, high expression of SNHG3 is an independent prognostic factor for glioma patients (Table 2). Furthermore, up-regulated SNHG3 predicted poor prognosis for glioma patients (Figure 1E). Such data indicated that SNHG3 might played as an oncogene in the progression of glioma.

**Figure 1:** Highly expressed SNHG3 predicts poor prognosis for glioma patients (**A**) The expression pattern of SNHG3 in glioma tissues and normal tissues of TCGA database was identified and analyzed. (**B**) qRT-PCR detected the level of SNHG3 in 60 pairs of glioma tissues and non-malignant tissues. (**C**) The expression condition, if SNHG3 in glioma tissues which was in different tumor stages, was examined with qRT-PCR. (**D**) The high expression of SNHG3 in glioma cells was determined by qRT-PCR. (**E**) Kaplan–Meier method analyzed the correlation between the expression of SNHG3 and patients’ overall survival. Error bars represented the mean ± SD of at least three independent experiments; *P<0.05, **P<0.01, ***P<0.001 vs. control group.

**Table 1:** Correlation between SNHG3 expression and clinical features of glioma patients (*n*=60)

Variable	SNHG3 expression		*P*-value
	Low	High	
**Age**			
<50	8	15	0.063
≥50	22	15	
**Gender**			
Male	11	15	0.297
Female	19	15	
**KPS**			
<80	23	8	<0.001***
≥80	7	22	
**Histopathology**			
Conventional	18	16	0.602
Chondriod	12	14	
**Invasion condition**			
Yes	23	11	0.002**
No	7	19	
**Tumor grade**			
I-II	24	11	0.001**
III-IV	6	19	

Low/high by the sample mean; Pearson χ^2^ test; **P<0.01, ***P<0.001 was considered statistically significant.

**Table 2:** Multivariate and univariate analysis of prognostic parameters in patients with glioma by Cox regression analysis

Variable	Category	Multivariate *P*-value	Univariate *P*-value
**Age**	<50	0.476	0.389
	≥50		
**Gender**	Male	0.240	0.290
	Female		
**KPS**	<80	0.492	0.011*
	≥80		
**Histopathology**	Conventional	0.198	0.210
	Chondriod		
**Invasion condition**	Yes	0.325	0.503
	No		
**Tumor grade**	I-II	0.008**	0.247
	III-IV		
**SNHG3 expression**	Low	0.001***	0.047
	High		

Proportional hazards method analysis showed a positive, independent prognostic importance of SNHG3 expression (*P*=0.001). *P<0.05, **P<0.01, ***P<0.001 was considered statistically significant.

### Down-regulated SNHG3 impairs cell proliferation through inducing cell cycle arrest and apoptosis

To clearly define how SNHG3 affected the growth of glioma, we prepared a series of functional assays with down-regulated SNHG3 in glioma cells and the transfection efficiency was obtained by using specific sh-RNA for SNHG3 (Figure 2A). It was observed that cell viability and proliferation rates were decreased a lot in cells transfected with sh-SNHG3, compared with the negative control (Figure 2B,C). Moreover, it was also observed that the knockdown of SNHG3 induced cell apoptosis and cell cycle arrest in G0/G1 phase (Figure 2D,E), implying that silenced SNHG3 impaired cell proliferation via triggering cell apoptosis and cell cycle arrest.

**Figure 2:** Silenced SNHG3 impairs cell proliferation via affecting cell cycle and apoptosis (**A**) qRT-PCR examined the expression of SNHG3 in cells transfected with sh-SNHG3. (**B** and **C**) MTT and colony formation assays were performed to measure the effect of silenced SNHG3 on cell proliferation. (**D** and **E**) Flow cytometry analyses were applied to examine the effect of silenced SNHG3 on cell cycle and apoptosis. Error bars represented the mean ± SD of at least three independent experiments; **P< 0.01 vs. control group.

### The effects of SNHG3 overexpression on cell proliferation, cell cycle distribution, and cell apoptosis

Above findings indicated that up-regulation of SNHG3 promoted glioma cell proliferation through affecting cell cycle distribution and cell apoptosis. Here, we designed gain-of-function assay to further demonstrate the oncogenic role of SNHG3 in glioma progression. The lowest expression of SNHG3 was observed in U251 cell, we enhanced the level of SNHG3 by transfecting pcDNA-SNHG3 overexpression vector. Forty-eight hours later, the best transfection efficiency was identified through comparing with empty vector. Next, MTT and colony formation assays were carried out in U251 cell transfected with pcDNA-SNHG3. As expected, cell proliferation was promoted by SNHG3 overexpression (Figure 3B,C). Consistent with loss-of-function assays, we applied flow cytometry analyses to analyze the effects of up-regulated SNHG3 on cell cycle distribution and cell apoptosis. Cell was gathered in S phase from G0/G1 phase (Figure 3D). Additionally, SNHG3 overexpression induced higher cell apoptosis rate (Figure 3E). All these findings helped us further confirm the oncogenic function of SNHG3 in glioma progression.

**Figure 3:** The effects of SNHG3 overexpression on cell proliferation, cell cycle distribution, and cell apoptosis (**A**) qRT-PCR examined the expression of SNHG3 in U251 cell transfected with pcDNA-SNHG3. (**B** and **C**) MTT and colony formation assays were performed to measure the effect of SNHG3 overexpression on cell proliferation. (**D** and **E**) Flow cytometry analyses were applied to examine the effect of SNHG3 up-regulation on cell cycle and apoptosis. Error bars represented the mean ± SD of at least three independent experiments; **P< 0.01 vs. control group.

### Down-regulated KLF2 and p21 were negatively correlated with SNHG3 in glioma tumorigenesis

It had been reported that KLF2 and p21 could participate in lncRNA-mediated tumorigenesis [15]. In order to differentiate whether KLF2 and p21 were also involved in SNHG3-mediated tumorigenesis in glioma, we examined the expressions of KLF2 and p21 in glioma tissues, exposing that both of the expressions of KLF2 and p21 were down-regulated in glioma tissues, in comparison with the normal ones (Figure 4A). Additionally, Spearman’s correlation analysis demonstrated that both KLF2 and p21 were negatively correlated with SNHG3 in glioma tissues (Figure 4B). In order to define the relationship among KLF2, p21 and SNHG3, we applied qRT-PCR and Western blot to detect the expression changes of KLF2 and p21 with the knockdown of SNHG3. It was discovered that both the mRNA and protein levels of KLF2 and p21 were enhanced after SNHG3 was impaired, which then were weakened slightly by the attenuation of KLF2 and p21 (Figure 4C–F), affirming the inverse association among the three genes above. These findings indicated that KLF2 and p21 might interact with SNHG3 in the tumorigenesis of glioma.

**Figure 4:** Down-regulated KLF2 and p21 are negatively associated with SNHG3 in glioma (**A**) qRT-PCR detected the expressions of KLF2 and p21 in glioma tissues. (**B**) Spearman’s correlation analysis determined the relationship between SNHG3 and KLF2 as well as between SNHG3 and p21. (**C**–**F**) Rescue assays were designed to further confirm the relationship between SNHG3 and KLF2/p21. Error bars represented the mean ± SD of at least three independent experiments; **P<0.01 vs. control group.

### SNHG3 epigenetically silences KLF2 and p21 through sponging with EZH2

To confirm the interaction of SNHG3 with KLF2 and p21, we first detected the expression of SNHG3 in nucleus and cytoplasm. As exhibited in Figure 5A, SNHG3 was mainly distributed in nucleus, indicating that SNHG3 regulated the glioma carcinogenesis at transcriptional level. It had been documented that KLF2 and p21 could be regulated by EZH2 [16,17]. So, we supposed that EZH2 may involve in the regulation of SNHG3/KLF2 and p21 pathway. It had been confirmed that the suppression of SNHG3 enhanced the KLF2 and p21 in Figure 4. Therefore, we next detected the effect of silenced EZH2 on KLF2 and p21, discovering that the knockdown of EZH2 also improved the mRNA and protein levels of KLF2 and p21 (Figure 5B,C). EZH2 is one member of polycomb group genes. In order to differentiate whether SNHG3 regulated the expressions of KLF2 and p21 via sponging with PRC2, we applied RIP assay and ensured that SNHG3 could bind to EZH2 (Figure 5D,E). Moreover, ChIP assays presented that EZH2 could directly bind to the promoter regions of KLF2 and p21, and then triggered H3K27me3 modification (Figure 5F). However, the silence of SNHG3 impaired the binding of EZH2 to the promoter regions of KLF2 and p21 (Figure 5G). Such results indicated that SNHG3 accelerated the malignancy of glioma through inhibiting the transcription of KLF2 and p21.

**Figure 5:** SNHG3 epigenetically silences KLF2 and p21 through sponging with EZH2 (**A**) Subcellular fractionation assay determined the location of SNHG3. (**B** and **C**) qRT-PCR and Western blot were applied to explore the effect of silenced EZH2 on the expressions of KLF2 and p21. (**D** and **E**) RIP detected the binding of SNHG3 to EZH2. (**F**) ChIP determined the binding of ZEH2 in the promoters of KLF2 and p21, and analyzed the H3K27me3 modification. (**G**) ChIP analyzed the effect of silenced SNHG3 on the binding of EZH2 to KLF2 and p21 promoters and on the H3K27me3 modification. Error bars represented the mean ± SD of at least three independent experiments; *P<0.05 and **P< 0.01 vs. control group.

### Regulation of expression of SNHC3, KLF2, and p21 affects the proliferation, cell cycle, and apoptosis

In order to proceed rescue assay, MTT assays were first employed in A172 cells to detect glioma cell proliferation ability. We discovered that the transfection of pcDNA-SNHG3 could greatly promote proliferation ability. However, the ability of glioma cell slightly declined when we transfected pcDNA-SNHG3+pcDNA-KLF2 and pcDNA-SNHG3+pcDNA-p21 into A172 cell (Figure 6A). With the help of flow cytometry, we measured the cell cycle and cell apoptosis. It was observed that the overexpression of SNHG3 inhibited cell apoptosis and cell cycle arrest in G2/M phase. When we added pcDNA-KLF2 or pcDNA-p21 into cell, cell apoptosis increased again and cell cycle more remained in S phase (Figure 6B,C). In brief, the cell proliferation was promoted by pcDNA-SNHG3, while were reduced again by adding pcDNA-KLF2 or pcDNA-p21.

**Figure 6:** Regulation of expression of SNHC3, KLF2, and p21 affects the proliferation, cell cycle, and apoptosis (**A**) MTT was performed to measure cell proliferation after co-transfection of pcDNA-SNHG3 and pcDNA-KLF2 or pcDNA-p21. (**B** and **C**) Flow cytometry analyses were applied to examine cell cycle and apoptosis after it subjected to the same co-transfection. Error bars represented the mean ± SD of at least three independent experiments; *P<0.05, **P<0.01 vs. control group.

## Discussion

The dysregulation of lncRNAs can provide cancers with a superiority for cellular growth through affecting epigenetic information, thus leading to uncontrolled tumor growth [18,19]. Effective regulation of cell survival and proliferation is important for tumorigenesis prevention and efficient cancer treatment [20]. Thereby, it may provide a novel insight for oncogenic mechanism to identify tumor-related lncRNAs as well as their clinical functions. LncRNA SNHG3 is a recently determined non-protein-coding RNA, and has just been analyzed in colorectal cancer and hepatocellular carcinoma [13,14]. It functions in glioma are unclear.

With Cys2/His2 zinc-finger domains, the Kruppel-like factor (KLF) family transcription factors can act as suppressors or activators in a cell type and promoter-dependent manner, and participate in cell differentiation and proliferation [21,22]. Some of the KLF family members can function as tumor suppressors, which is attributed to the inhibitory roles in proliferation and migration, and to the apoptosis induction [23,24]. As one of KLF families, KLF2 is down-regulated in various cancers with tumor-suppressor characteristics including KRAS-mediated inhibition of cell proliferation [25–27]. What’s more, it has been acknowledged that the expression of KLF2 and p21-mediated suppressive traits of KLF2 can be attenuated by EZH2 [17]. Although multiple genes have been reported to be capable of interacting with KLF2 and p21, such as GHET1 and KLF2 in hepatocellular carcinoma [28], SNHG15 and KLF2 in pancreatic cancer [29], HOXA-AS2, p21 and KLF2 in colorectal cancer [15], the interaction among SNHG3, KLF2 and p21 is still masked.

In the present study, we determined the expression level of SNHG3 in glioma tissues and cells and evaluated the effect of SNHG3 expression on the prognosis of glioma patients. The functional assays were applied to define the effects of SNHG3 on the biological behaviors in glioma including cell proliferation, cell cycle, and apoptosis. It was revealed that SNHG3 was much more enriched in glioma tissues and cell lines than in normal ones. Furthermore, loss-of-function experiments indicated that the knockdown of SNHG3 repressed cell proliferation, led to cell cycle arrest, and induced apoptosis. The mechanistic assays disclosed that SNHG3 facilitated the malignant progression of glioma through epigenetically repressing KLF2 and p21 via recruiting EZH2 to the promoter of KLF2 and p21. Generally, it was exposed that SNHG3 might function as an oncogene in glioma and could be explored as a potential prognostic biomarker and therapeutic target for glioma.

## Abbreviations

EZH2: enhancer of zeste homolog 2
KLF: Kruppel-like factor
lncRNA: long non-coding RNA
ncRNA: non-protein-coding RNA
RIP: RNA immunoprecipitation
SHNG3: small nucleolar RNA host gene 3
